The article "Structural simulation of adenosine phosphate via plumbagin and zoledronic acid competitively targets JNK/Erk to synergistically attenuate osteoclastogenesis in a breast cancer model" was retracted in 2019. Reasons: errors in the images; unreliable data; unreliable images.

# Structural simulation of adenosine phosphate via plumbagin and zoledronic acid competitively targets JNK/Erk to synergistically attenuate osteoclastogenesis in a breast cancer model

**DOI:** 10.1038/cddis.2016.11

**Published:** 2016-02-11

**Authors:** H Qiao, T-y Wang, Z-f Yu, X-g Han, X-q Liu, Y-g Wang, Q-m Fan, A Qin, T-t Tang

**Affiliations:** 1 Shanghai Key Laboratory of Orthopaedic Implants, Department of Orthopaedic Surgery, Shanghai Ninth People's Hospital, Shanghai Jiao Tong University School of Medicine, Shanghai, China; 2 Shanghai Key Laboratory of Orthopaedic Implants, Department of Pharmacy, Shanghai Ninth People's Hospital, Shanghai Jiao Tong University School of Medicine, Shanghai, China

## Abstract

The treatment of breast cancer-induced osteolysis remains a challenge in clinical settings. Here, we explored the effect and mechanism of combined treatment with zoledronic acid (ZA) and plumbagin (PL), a widely investigated component derived from *Plumbago zeylanica*, against breast cancer-induced osteoclastogenesis. We found that the combined treatment with PL and ZA suppressed cell viability of precursor osteoclasts and synergistically inhibited MDA-MB-231-induced osteoclast formation (combination index=0.28) with the abrogation of recombinant mouse receptor activator of nuclear factor-*κ*B ligand (RANKL)-induced activation of NF-*κ*B/MAPK (nuclear factor-*κ*B/mitogen-activated protein kinase) pathways. Molecular docking suggested a putative binding area within c-Jun N-terminal kinase/extracellular signal-regulated kinase (JNK/Erk) protease active sites through the structural mimicking of adenosine phosphate (ANP) by the spatial combination of PL with ZA. A homogeneous time-resolved fluorescence assay further illustrated the direct competitiveness of the dual drugs against ANP docking to phosphorylated JNK/Erk, contributing to the inhibited downstream expression of c-Jun/c-Fos/NFATc-1 (nuclear factor of activated T cells, cytoplasmic, calcineurin-dependent 1). Then, *in vivo* testing demonstrated that the combined administration of PL and ZA attenuated breast cancer growth in the bone microenvironment. Additionally, these molecules prevented the destruction of proximal tibia, with significant reduction of tartrate-resistant acid phosphatase (TRAcP)-positive osteoclast cells and potentiation of apoptotic cancer cells, to a greater extent when combined than when the drugs were applied independently. Altogether, the combination treatment with PL and ZA could significantly and synergistically suppress osteoclastogenesis and inhibit tumorigenesis both *in vitro* and *in vivo* by simulating the spatial structure of ANP to inhibit competitively phosphorylation of c-Jun N-terminal kinase/extracellular signal-regulated kinase (JNK/Erk).

The article "Structural simulation of adenosine phosphate via plumbagin and zoledronic acid competitively targets JNK/Erk to synergistically attenuate osteoclastogenesis in a breast cancer model" was retracted in 2019. Reasons: errors in the images; unreliable data; unreliable images.

Recent decades have witnessed an increasing number of patients diagnosed with malignant breast cancer that includes serious metastatic bone destruction and decreased life expectancy.^1, 2, 3^ In these patients, cancer-associated bone tissues endure a series of cancer-induced pathological processes,^4^ which are triggered by the excessive activation of bone absorption by osteoclast cells,^5^ and therefore contributing to the establishment of distant osteolytic lesions and influencing the normally well-balanced skeletal physiological functionality and structural integrity. Bisphosphonates such as zoledronic acid (ZA), which constitute the bone-modifying agents, have demonstrated efficacy in reducing osteoclast-induced bone loss in metastatic cancer patients.^6^ However, the actual pharmacological efficacy of ZA against tumorigenesis has remained debatable, with the drug displaying varying cytotoxicity against human breast cancer cells and inevitable side effects such as severe osteonecrosis of the jaw (ONJ), atypical fractures and others.^7, 8, 9, 10, 11^ As a result, combined treatment with ZA and other pharmacological reagents or nutraceuticals, such as cisplatin, doxorubicin, gemcitabine and camellia sinensis,^12, 13, 14^ in various cancers was introduced to potentiate the effects of chemotherapy.

Our previous study exploited combined administration of ZA with one widely analyzed medical compound, plumbagin (PL), which is derived from the historical Chinese plant *Plumbago zeylanica*, to investigate the combined *in vitro* effects against MDA-MB-231SArfp human breast cancer cells.^15^ This work showed that combined treatment was able to repress synergistically breast tumor malignancy *in vitro* through modulation of Notch-1-Bcl-2. However, it remains unclear whether the combination of PL with ZA will have synergistic effects against osteoclastogenesis. So far, we have demonstrated that PL and ZA could synergistically suppress cancer-induced osteoclastogenesis and tumorigenesis both *in vitro* and *in vivo*. More importantly, we found that the molecular structure of the combined drugs was able to mimic an ANP molecule, thereby competitively inhibiting phosphorylation of a targeted protein kinase. These results suggest a potentially novel mechanism of drug combination against cancer-associated osteoclastogenesis that can be applied to other research fields.

## Results

### Combined treatment with PL and ZA synergistically inhibited the viability of osteoclast precursor cells

The effects of drug treatment on the viability of RAW264.7 osteoclast precursor monocytes were initially determined. Treatment with PL at concentrations ranging from 5 to 20 *μ*M along with administration of ZA in concentrations from 12.5–100 *μ*M significantly repressed the viability of RAW264.7 cells from 24 to 96 h. Additionally, the toxicity of ZA against precursor osteoclasts increased over time. We found an additional effect at 6.25 *μ*M from 48 to 72 h and at 3.125 *μ*M at 96 h treatment (Figures 1a and b). The half-maximal inhibitory concentration (IC_50_) at 48 and 72 h was calculated as 12 and 7.1 *μ*M in the PL group and 227 and 32 *μ*M in the ZA group, respectively. When RAW264.7 cells were simultaneously treated with PL and ZA, 5, 10 and 20 *μ*M of PL synergistically increased the growth inhibitory effects of almost every concentration of ZA after 24–96 h when compared with treatment with ZA alone. Meanwhile, 2.5 *μ*M of PL potentiated the cytotoxicity of ZA at the later time point (96 h). No obvious synergistic potential was found with the combination of 5, 10 or 20 *μ*M of PL with 100 *μ*M of ZA from 48 to 96 h or with 50 *μ*M of ZA at 96 h. Similarly, 25, 50 and 100 *μ*M of ZA enhanced the repressive effects of low concentrations of PL (1.25 and 2.5 *μ*M at 24 h and 1.25, 2.5 and 5 *μ*M at all observed time points). Additionally, 12.5 *μ*M of ZA was instrumental in the proliferative suppression by PL at concentrations of 2.5 and 5 *μ*M at 72 h and 1.25, 1.55 and 5 *μ*M at 96 h. No evident synergism (Syn) was found when RAW264.7 cells were treated with a combination of 12.5–100 *μ*M of ZA and 5 *μ*M of PL at 24 h, or 10–20 *μ*M of PL from 24 to 96 h (Figures 1c and d).

The article "Structural simulation of adenosine phosphate via plumbagin and zoledronic acid competitively targets JNK/Erk to synergistically attenuate osteoclastogenesis in a breast cancer model" was retracted in 2019. Reasons: errors in the images; unreliable data; unreliable images.

The fraction affected-combination index (Fa-CI) plot and fraction affected-dose-reduction index (Fa-DRI) plot (Figure 1e) generated by the Compusyn software were created to elucidate the potency of Syn between PL and ZA. The CI values were 0.28 and 0.83 (<1) when Fa equaled 0.5 and 0.75, respectively, revealing an explicit synergistic antiosteoclastogenesis potential in the combination of PL and ZA. The DRI values were 14.7, 4.68 and 7.39, 1.45 (>1) for PL and ZA when the Fa level was 0.5 and 0.75, illustrating the therapeutic pharmacological advantages of the combination, which could have practical clinical applications.

### PL and ZA synergistically inhibited MDA-MB-231-induced osteoclastogenesis *in vitro*

Breast cancer cells secrete recombinant mouse receptor activator of nuclear factor-*κ*B ligand (RANKL) to facilitate osteoclast formation.^16^ Both bone marrow-derived monocytes (BMMs) stimulated with RANKL (Figure 2A) and human peripheral blood mononucleated cells (hPBMCs) stimulated with conditioned medium (CM) from MDA-MB-231 human breast cancer cells (Figure 2B) were able to develop significant, multinucleated osteoclasts. In contrast, PL and ZA alone significantly inhibited RANKL-induced osteoclastogenesis of BMMs in a concentration-dependent manner. hPBMCs treated with CM containing PL and ZA demonstrated a decreased number and area of TRAcP-positive cells dose-dependently. Moreover, combined treatment synergistically suppressed the differentiation of precursor osteoclasts (BMMs and hPBMCs) by both RANKL- and MDA-MB-231-induced activation, as illustrated by the facts that dual treatments using low concentrations of the drugs (2.5 *μ*M PL with 0.3 *μ*M ZA and 1.25 *μ*M PL with 0.7 *μ*M ZA) were able to completely block formerly active osteoclastogenesis.

The article "Structural simulation of adenosine phosphate via plumbagin and zoledronic acid competitively targets JNK/Erk to synergistically attenuate osteoclastogenesis in a breast cancer model" was retracted in 2019. Reasons: errors in the images; unreliable data; unreliable images.

### Synergistic treatment with PL and ZA repressed RANKL-induced activation of the NF-*κ*B and MAPK pathways

Activation of the nuclear factor-*κ*B (NF-*κ*B) cascade is marked by decreased expression of I*κ*B*α* and increased production of p-I*κ*B*α* and p-p65, without changes in the levels of p65 or the upstream I*κ*B kinase (IKK) complex.^17, 18^ The RANKL-induced activation of p-I*κ*B*α* and p-p65, as well as the degradation of I*κ*B*α*, was inhibited by treatment with PL (10 *μ*M), ZA (50 *μ*M) and Syn (PL 10 *μ*M plus ZA 50 *μ*M) (Figure 3A). Moreover, JNK, extracellular signal-regulated kinase 1/2 (Erk-1/2) and p38 are considered to be the main subfamilies of mitogen-activated protein kinases (MAPKs), with evidence showing that the phosphorylated MAPKs could contribute to differentiation toward mature osteoclasts in precursor cells.^17^ Intervention with PL (10 *μ*M), ZA (50 *μ*M) and Syn (PL 10 *μ*M plus ZA 50 *μ*M) attenuated the RANKL-stimulated phosphorylated JNK and Erk, whereas ZA and Syn administration suppressed RANKL-induced phosphorylated p38 (Figure 3B). Indeed, based on western blots, the Syn group appeared to exert the most evident inhibitory effects on RANKL-induced NF-*κ*B and MAPK activation when compared with individual treatment. The inhibitory effects of synergistic administration were most evident upon JNK/Erk phosphorylation, which were thus used for further mechanism analysis.

### Interaction between dual drugs and JNK-1/Erk-1

Interestingly, the two- and three-dimensional structures of PL, ZA and ANP showed that, to a large extent, the combination of PL with ZA could simulate the complanate and stereostructure of ANP (Figure 4A). The combination of PL with ZA could embed properly into the ANP binding pockets of JNK-1 and Erk-1 kinase using a spatial structure similar to that of ANP. Specifically, the dual drugs linked to MET111, LEU110, GLN37, LYS153, ASP169 and GLU73 of JNK-1 kinase and ASP124, MET126, LYS169, ASN172 and ASP185 of Erk-1 kinase (Figure 4B). The combined drugs occupied the ANP binding sites, thereby competitively blocking ANP from binding its kinase and attenuating the ANP-dependent phosphorylated forms.

The article "Structural simulation of adenosine phosphate via plumbagin and zoledronic acid competitively targets JNK/Erk to synergistically attenuate osteoclastogenesis in a breast cancer model" was retracted in 2019. Reasons: errors in the images; unreliable data; unreliable images.

### Competition with ANP via structural simulation of PL and ZA against phosphorylation of JNK/Erk

We next performed homogeneous time-resolved fluorescence (HTRF) assays to investigate the competitiveness of individual drug and dual drugs against ANP bindings towards JNK-1 and Erk-1 kinases. Based on the criterion mentioned above, an optimal enzyme reaction condition of 0.11 *μ*M for 60 min against JNK-1 and Erk-1 was initially illustrated (Figure 4C). Next, the drug's competitiveness with ANP was measured by HTRF assay using inhibitor IC_50_ values over a scale of ANP concentrations. If drugs failed to outcompete ANP binding, no change in IC_50_ would be expected. Along with the increase of JNK-1/Erk-1 ANP *K*_m_ from 1*K*_m_ to 9*K*_m_, the IC_50_ curves of PL alone moved insignificantly with faintly increase of IC_50_ from 0.2477 to 0.2929 and 0.2420 to 0.3252 *μ*M, respectively. Besides, the increase of JNK-1/Erk-1 ANP *K*_m_ from 1*K*_m_ to 9*K*_m_ also failed to contribute to the significant right shift of the IC_50_ curves of ZA alone with negligible IC_50_ changes from 4.491 to 6.111 and 26.20 to 29.28 *μ*M, respectively (Figure 4D). However, we found that with the increase of JNK-1 ANP *K*_m_, the IC_50_ curve of the dual drugs shifted to the right significantly and the values increased at least 16-fold from 0.264 to 4.362 *μ*M. Similarly, along with the increase of Erk-1 ANP *K*_m_, the IC_50_ curve shifted to the right remarkably and the values increased at least twofold from 0.4411 to 1.195 *μ*M (Figure 4E). Such results showed that to achieve the same level of phosphorylation, a greater dosage of the dual drugs was required for an increased number of ANP concentrations, indicating direct competition of the dual drugs with ANP for binding to JNK-1 and Erk-1 kinase.

Furthermore, the downstream expressions of c-Jun, c-Fos and NFATc-1 (nuclear factor of activated T cells, cytoplasmic, calcineurin-dependent 1), which should be activated following JNK/Erk phosphorylation, were inhibited significantly in the presence of dual drugs (Figure 4F). This result indicated that the dual drugs were able to target the upstream kinase and abrogate phosphorylation, thereby decreasing the levels of downstream functional proteins (Figure 5).

### Combined treatment with PL and ZA synergistically attenuates the growth of breast cancer cells in the bone microenvironment

A noninvasive *in vivo* imaging system (IVIS) revealed that all three drug interventions significantly decreased both fluorescence intensity and tumor size compared with the vehicle control group. Representative specimens from each individual group were presented (Figure 6A) to demonstrate the significant inhibition exerted by various drugs on growth of MDA-MB-231SArfp cells in a local bone microenvironment. Specifically, both PL and ZA treatment alone reduced tumorigenesis by 1–2 weeks and decreased tumor volume by 33–50% compared with vehicle-treated mice. Moreover, a marked postponement of tumor initiation until the fourth week, along with a reduction in tumor size by 60–68%, was witnessed in the combination group. This result signified a synergistic effect against the establishment and development of metastatic mammary tumors through administration of combined drugs *in vivo* (Figure 6B). From the fourth week on, the nude mice from the vehicle, PL and ZA groups experienced a marked surge in tumor development, whereas the mice treated with the combined drugs retained a relatively low level of tumor intensity that lasted into the end of the 6-week observation, implicating an effective antitumor effect of synergistic treatment with PL and ZA. A correlation (*γ*^2^=0.9673) to determine the connection between fluorescence intensity and tumor volume was also found in the 6-week observation. All of the experimental animals showed stability in body weight and regular activity (data not shown), demonstrating that treatment with neither individual nor combined drugs resulted in any evident toxicity for normal cells.

The article "Structural simulation of adenosine phosphate via plumbagin and zoledronic acid competitively targets JNK/Erk to synergistically attenuate osteoclastogenesis in a breast cancer model" was retracted in 2019. Reasons: errors in the images; unreliable data; unreliable images.

### Combined treatment with PL and ZA synergistically suppressed breast cancer cell-induced osteolytic lesions *in vivo*

X rays showed that osteolytic damage was not present in any of the sham-treated tibiae, whereas cancer-induced osteolysis, including complete destruction of proximal tibia and knee joint, developed in vehicle-treated mice. Nonetheless, both individual and combined treatments were capable of arresting bone erosion and maintaining the intact structure of the knee joint (Figure 7A). Furthermore, as shown in representative *μ*CT graphs (Figures 7B and C), treatments with PL, ZA and Syn were able to prevent cancer-induced osteolysis and maintain fundamental integrity of the knee joint. Quantification of bone parameters revealed that both PL and ZA attenuated the extensive lytic lesions, with a clear increase of trabecular bone volume/tissue volume (BV/TV) and Cor. BV/TV (Figure 7D), which were the key indicators of bone mass. Additionally, combined treatment exhibited a synergistic effect on tumor-induced osteolysis, a result that was confirmed by the higher levels of BV/TV compared with the individual intervention.

The article "Structural simulation of adenosine phosphate via plumbagin and zoledronic acid competitively targets JNK/Erk to synergistically attenuate osteoclastogenesis in a breast cancer model" was retracted in 2019. Reasons: errors in the images; unreliable data; unreliable images.

### Histology of osteoclast activity of proximal tibia specimens

In sections from vehicle-treated mice, routine hematoxylin and eosin (H&E) staining (Figure 8A) revealed that metaphyseal bones were nearly destroyed with the apparent disappearance of the basic trabecular architecture. However, H&E slides from samples treated with individual drugs exhibited a rescued metaphysis and a multitude of trabecular systems. This phenotype was especially notable in ZA-treated tumor-bearing nude mice. Moreover, sections from mice treated simultaneously with both drugs showed not only an almost entirely integrated knee configuration but also an intact metaphysis including a wealth of preserved trabecular network. Next, TRAcP staining (Figure 8B) revealed numerous mature TRAcP-positive osteoclasts in slides prepared to show trabecular structure from vehicle-treated legs (27–31%). A lower proportion of stained osteoclasts were observed in PL- and ZA-treated mice (8–13% and 5–8%, respectively). Significantly, the lowest positive rate of TRAcP staining was found among sections from the Syn group of nude mice (1–3%), with no red-stained cells detected within trabecular bone. This result led to the conclusion that synergistic treatment could not only attenuate the process of tumorigenesis but also inhibit the progression of cancer-induced osteoclastogenesis *in vivo*.

### Immunohistochemistry of tumor specimens

Immunohistochemistry for red fluorescent protein (RFP) protein (Figure 8C) confirmed the successful implantation of MDA-MB-231SArfp cells in targeted tumor-bearing tibiae. Quantitative results revealed no significant difference between the vehicle, PL and ZA groups. However, there was a significant difference in the Syn group, which further demonstrated a restricted expression of RFP protein (34–42%) in the bone microenvironment when treated with both PL and ZA. Additionally, Ki-67 (Figure 8D) and TUNEL (transferase-mediated dUTP biotin nick-end labeling) (Figure 8E) immunohistochemistry demonstrated that treatment with both PL and ZA reduced the percentage of Ki-67-positive cells and increased the proportion of TUNEL-positive cells compared with vehicle treatment (*Ki-67*-positive cells were 36–45% in vehicle-treated group, 18–23% in PL-treated group, 21–26% in Za-treated group; *TUNEL*-positive cells were 6–10% in vehicle-treated group, 26–33% in PL-treated group, 18–23% in Za-treated group). This result helps to explain the advantageous antitumoral pharmacologic capabilities of the drugs against establishment of MDA-MB-231SArfp cells *in vivo*. More importantly, a minimal proportion of Ki-67-positive cells and a multitude of TUNEL-positive cells were observed in slides from nude mice treated with both drugs (*Ki-67*-positive cells were 8–13% in dual drugs-treated group, *TUNEL*-positive cells were 37–42% in dual drugs-treated group). All of above results demonstrated a potentiated synergistic efficacy against tumorigenesis through combined treatment with PL and ZA in an intratibial nude mouse model of breast cancer.

The article "Structural simulation of adenosine phosphate via plumbagin and zoledronic acid competitively targets JNK/Erk to synergistically attenuate osteoclastogenesis in a breast cancer model" was retracted in 2019. Reasons: errors in the images; unreliable data; unreliable images.

## Discussion

In this study, PL was used as an effective adjuvant treatment in reinforcing the ZA-modulated antiosteoclastogenesis and antitumorigenesis both *in vitro* and *in vivo* by simulating ANP structure synergistically to target competitively phosphorylation of JNK/Erk, thereby decreasing breast cancer-induced osteoclast formation. PL has been proven to attenuate malignant revolution in various cancer categories^2, 15, 19, 20, 21, 22^ and suppress the progress of atherosclerosis, inflammation, malaria, immune response and microbial infection, and so on.^23, 24, 25, 26^ However, no exiting study shows the combinative effects of PL with other reagent against cancer-induced osteolysis. Herein, we pioneered to unravel that PL was capable of synergizing anti-bone destruction impacts with one commonly used pharmacologic strategy both *in vitro* and *in vivo*, indicating a potential promising application of PL clinically.

Currently, bisphosphonates such as ZA is ubiquitously administered intravenously to treat early bone metastatic carcinomas in clinic by inhibiting osteoclast-mediated bone resorption.^27, 28^ ZA inhibits crucial enzymes of the mevalonate pathway, including farnesyl pyrophosphate synthase and geranylgeranyl pyrophosphate synthase, contributing to the repressive post-translational prenylation of GTPases signaling, thereby triggering the apoptosis of osteoclasts.^29, 30^ Nonetheless, the utilization of ZA was largely restrained owing to the varying cytotoxicity and unavoidable side effects, mainly involved gastrointestinal symptoms, muscle pain, atypical fractures, ONJ and ocular inflammation,^31^ intriguing a number of researchers into exploring the best optimization of the usage of ZA. Unsurprisingly, the synergistic treatment strategy of ZA with other drug occurred, implicating that the actual dosage of ZA could be diminished to achieve regular or even better efficacy, leading to the alleviation of cytotoxicity and side effects. In a rat model of postmenopausal osteoporosis, combination therapy of alfacalcidol with ZA demonstrated significant preserved trabecular microstructure and cortical bone density with decreased serum TRAcP level than alfacalcidol or ZA alone.^32^ Yu *et al.*^33^ illustrated that the combination of ZA with everolimus was able to relieve the cancer-induced bone devastation greatly than individual treatment, as further assessed by the significant decreased layer of crosslinked NTX, the biomarker of osteolytic cell activity in combination group. Our results showed that the combination of PL with ZA decreased precursor osteoclast viability synergistically with CI value <1 and DRI (PL), DRI (ZA) values >1. Furthermore, breast cancer cells secrete RANKL to facilitate osteoclast formation both *in vitro* and *vivo.*^16^ The administration of dual drugs inhibited osteoclast formation significantly compared with individual PL or ZA when BMMs and hPBMCs were induced with RANKL directly and MDA-MB-231, respectively.

The article "Structural simulation of adenosine phosphate via plumbagin and zoledronic acid competitively targets JNK/Erk to synergistically attenuate osteoclastogenesis in a breast cancer model" was retracted in 2019. Reasons: errors in the images; unreliable data; unreliable images.

During osteoclast formation, the induction of osteoclast precursors with RANKL is thought to bind with RANK, the signaling adaptor molecule, and activate the phosphorylation of I*κ*B*α* and its subsequent degradation,^34, 35^ followed by increased translocation and phosphorylation of downstream p65,^36^ altogether contributing to the activation of the NF-*κ*B pathway. Also, subunits of MAPKs (JNK, Erk-1/2 and p38) have a pivotal role during osteoclastogenesis.^37, 38^ Downregulation of Erk inhibits the merging of osteoclast precursors, suppression of JNK impedes RANKL-stimulated osteoclastogenesis^39, 40, 41^ and activation of p38 contributes greatly to the early maturation of osteoclasts.^42^ NF-*κ*B and MAPK pathways that comprise distinct kinases require the active communication between functional proteins with ANP to provide phosphate group^43, 44^ for the sake of phosphorylating substrates and displaying regulative mechanism during osteoclast formation.^45, 46^ Consequently, kinase inhibitors that competitively block the binding of ANP to the so-called ‘deep pocket' emerged, altering the conformation of targeted enzymes into enzymatically silent states^47, 48^ and impacting subsequent bioactivities.^49, 50^ In our study, the major structural features of PL and ZA are naphthaline (10-atom ring) and imidazole (5-atom ring), respectively. Similarly, the basic structure of ADP is comprised of one 9-atom ring and one 5-atom ring, which suggest that the combination of PL with ZA might be able to simulate ANP, thus linking the drugs to the binding sites of kinases. Three-dimensional modeling confirmed our hypothesis, revealing that the combined drugs were capable of mimicking the stereostructure of ANP. Here, we first proposed that the combination of PL with ZA was able to serve as ANP inhibitor by simulating ANP structure to compete the active binding with JNK/Erk, leading to the potent inhibitory effects of breast cancer-associated osteoclast formation.

Undoubtedly, the progresses of tumor, microbial infection and inflammatory bone diseases are ATP-dependent diseases that require the active participation of ATP. Previous researches indicated that the combination of two widely used pharmacological drugs could influence the generation and transportation of ATP, decreasing the exploitation of ATP instead of individual treatment, leading to a synergistic effects against cancer cells, microbial infections and chronic arthritis.^51, 52, 53^ Therefore, we consider that the combinative treatment of PL with ZA can be applied in the treatment of tumor, microbial infection and inflammatory bone diseases by inhibiting ATP activities, which require future in-depth work.

The article "Structural simulation of adenosine phosphate via plumbagin and zoledronic acid competitively targets JNK/Erk to synergistically attenuate osteoclastogenesis in a breast cancer model" was retracted in 2019. Reasons: errors in the images; unreliable data; unreliable images.

As the intratibiae model of breast cancer closely re-establishes the progress of breast cancer-induced osteolysis,^54^ we chose such model to assess the synergistic effects of PL with ZA *in vivo*. Both osteoclastogenesis and tumorigenesis were significantly inhibited after administration of dual drugs compared with individual treatment, as illustrated with results from IVIS, X-ray, *μ*CT and histologic analysis. Nonetheless, the intratibiae breast cancer model failed to reconstruct the malignant metastasis from mammary tissues to distant skeletal system. Therefore, it was difficult to evaluate the antimetastasis effect of dual drugs, which demanded subsequent research. Moreover, the actual effectiveness of chemotherapy is limited owing to the resistance of target cells to treatment reagents, which urge to develop carrier-based site-specific delivery of chemotherapeutic drugs. Hence, a novel nanodelivery system and bone-targeted administration of PL conjugated with ZA would be an attractive strategy for treating bone metastases of breast cancer.^55, 56^

In conclusion, the combined treatment of PL with ZA suppressed the formation of cancer-induced osteoclastogenesis and tumorigenesis synergistically both *in vitro* and *in vivo.* Synergistic treatment with PL and ZA attenuated RANKL-stimulated activation of NF-*κ*B and MAPK signaling pathways during osteoclast formation through structural simulation of ANP to target competitively phosphorylation of JNK/Erk.

## Materials and Methods

### Materials and main reagents

The human breast cancer cell subline MDA-MB-231SArfp, which has a tendency to colonize and grow within the bone microenvironment, was generated as described previously.^57^ MDA-MB-231 and RAW264.7 cells were purchased from American Type Culture Collection (Rockville, MD, USA). MDA-MB-231SArfp, MDA-MB-231, RAW264.7, primary BMMs and hPBMCs were cultured with *α*-MEM medium (Hyclone, Logan, UT, USA) containing 10% fetal bovine serum (FBS; Hyclone). PL and ZA were purchased from Sigma-Aldrich (St. Louis, MO, USA). The combined treatment with ZA and PL *in vivo* and *in vitro* consisted of equal volumes of both drugs. RANKL and macrophage colony-stimulating factor (MCSF) were purchased from PeproTech (Rocky Hill, NJ, USA). The specific primary and second antibodies listed below were purchased from Cell Signaling Technology (Danvers, MA, USA) and Abcam (Cambridge, UK).

The article "Structural simulation of adenosine phosphate via plumbagin and zoledronic acid competitively targets JNK/Erk to synergistically attenuate osteoclastogenesis in a breast cancer model" was retracted in 2019. Reasons: errors in the images; unreliable data; unreliable images.

### Cell viability assay

The effects of various PL and ZA treatments on the viability of RAW264.7 cells were measured using the Cell Counting Kit-8 method.^58, 59^ The control groups were administered a vehicle reagent, whereas the PL and ZA groups were treated with corresponding drugs at varying concentrations for 24–96 h. Additionally, the synergistic groups were treated with equivalent ratios of PL and ZA at the required combined concentrations. The optical density at 450 nm was determined with a microplate reader (Thermo Electron Corp., Waltham, MA, USA). Experiments were repeated independently at least three times.

### Analysis of Syn

CompuSyn software (Combosyn Inc, Cambridge, MA, USA) was used to analyze the synergistic effects of PL and ZA according to a previous report^60^ and based on the median effect principle described by Chou and Talalay.^61^ Different Fa levels were indicative of different growth inhibitory effects (a range of Fa levels from 0.05 to 0.9 demonstrated a 5–90% inhibition of growth). The CI represents the pharmacological interaction between PL and ZA (CI<1, synergistic effect; CI=1, additive effect; CI>1, antagonistic effect). The DRI indicates the fold change of dose inhibition induced by synergistic administration relative to treatment with individual drugs at the required effector level. DRI>1 represented therapeutic significance showing the reduced side effects caused by either combination of drugs in normal cells. The Fa-CI and Fa-DRI plot signified the factual synergistic index at disparate suppressive extents by computerized operations.

### Preparation of CM from human breast cancer cells

Human breast cancer MDA-MB-231 cells (1 × 10^6^ cells) were seeded in T75 culturing flask with *α*-MEM medium supplemented with 10% FBS at 37 °C. Upon reaching nearly complete confluence, the medium was changed into serum-free *α*-MEM medium. After further incubation of 24 h, the medium as CM was collected and frozen at −20 °C.

### Isolation of hPBMCs

The isolation of hPBMCs was accomplished from healthy human peripheral blood with Ficoll density gradient centrifugation according to previous report.^62, 63^ Briefly, anticoagulated peripheral blood from healthy human donor was diluted with an equal volume of RPMI-1640 culturing medium (Hyclone). The diluted peripheral blood was layered over 20 ml of Ficoll solution (TBD science, Tianjin, China) and centrifuged horizontally at 2000 r.p.m. for 20 min at room temperature. The intermediate layer of hPBMCs was carefully removed with 1 ml syringe and washed with RPMI-1640 medium two times by centrifugation at 1500 r.pm. for 10 min. Harvested hPBMCs were cultured with *α*-MEM medium supplemented with 10% FBS and 60 ng/ml MCSF at 37 °C, 5% CO_2_.

The article "Structural simulation of adenosine phosphate via plumbagin and zoledronic acid competitively targets JNK/Erk to synergistically attenuate osteoclastogenesis in a breast cancer model" was retracted in 2019. Reasons: errors in the images; unreliable data; unreliable images.

### Assessment of cancer-associated osteoclastogenesis *in vitro*

BMMs were harvested from the tibiae and femur of 6-week-old C57 mice and incubated in *α*-MEM medium supplemented with 10% FBS and 30 ng/ml MCSF. MCSF has a vital role during proliferation of precursor osteoclast cells, whereas RANKL contributes greatly to the differentiation and absorptive functionality of osteoclasts.^64, 65, 66^ After harvest and transplantation into 96-well plates, BMMs were treated with either PL or ZA alone or various PL and ZA combinations containing 30 ng/ml MCSF and 50 ng/ml RANKL. For CM experiment, hPBMCs were seeded and added with CM containing 60 ng/ml MCSF and drug alone or varying combinations. After further incubation, TRAcP staining was performed on precursor osteoclast cells and mature osteoclast cells. TRAcP-positive multinucleated cells containing at least three nuclei were classified as mature osteoclasts. Experiments were repeated independently at least three times.

### Western blotting

RAW264.7 cells were seeded in 6-well plates at a density of 6 × 10^5^ cells per well overnight without drugs. After reaching 90% confluence, *α*-MEM medium lacking FBS and containing no drug, 10 *μ*M PL, 50 *μ*M ZA or 10 *μ*M PL plus 50 *μ*M ZA was added to the relevant wells for 4 h serum starvation. Then, starved RAW264.7 cells were treated with RANKL at a concentration of 50 ng/ml for 20 min. After the indicated time point, proteins were extracted for western blotting and visualized with an Odyssey Infrared Imaging System (LI-COR, Biosciences, Lincoln, NE, USA).

### Molecular docking

To investigate the potential docking sites of the dual drugs to the ANP binding pockets of JNK-1/Erk-1, which are the kinases upstream of c-Jun/c-Fos/NFATc-1, three-dimensional homology models of mouse JNK-1/Erk-1 kinase domains were established with Modeler 9.12 using the architectures of human JNK-1/Erk-1 as templates. The stereochemical constructs of JNK-1/Erk-1 were confirmed with PROCHECK. MolConverter and MarvinSketch were used to generate and refine the spatial coordinates for the drugs. The combined drugs were linked to ANP docking pockets in both JNK-1 and Erk-1 by the Lamarckian genetic algorithm based on AutoDock and AutoDock Vina.^67^ The resulting molecular modeling figures of binding activities were prepared with PyMOL Visualization Software (Schrödinger LLC, New York, NY, USA).

The article "Structural simulation of adenosine phosphate via plumbagin and zoledronic acid competitively targets JNK/Erk to synergistically attenuate osteoclastogenesis in a breast cancer model" was retracted in 2019. Reasons: errors in the images; unreliable data; unreliable images.

### HTRF assay

The HTRF assay was performed as reported previously^68, 69^ with minor adjustments. Briefly, substrates of JNK-1 and Erk-1 (Life, Carlsbad, CA, USA) were mixed and incubated with corresponding kinases to explore the optimal enzyme conditions with varying reaction times and concentrations. The criteria of enzyme optimization were (1) the highest slope indicating the widest reaction window and the most sensitive reaction condition to guarantee that the end point of an individual reaction was within the linear kinetic curve and (2) the restricted amount of enzymes. Then, the apparent ANP *K*_m_ for each kinase was determined^70^ (*K*_m_is the Michaelis constant for ANP) (excitation wavelength: 320 nm; emission wavelength: 620 nm). A volume of 2.5 *μ*l of drugs, containing 10 *μ*M PL, 50 *μ*M ZA or 10 *μ*M PL plus 50 *μ*M ZA at equal volumes, was mixed and supplemented with 2.55 *μ*l ATP/well (Sigma, St. Louis, MO, USA) and 5 *μ*l/well of substrate and kinase mixture to start the enzymatic steps. This reaction was carried out at room temperature for 1 h. The 10 *μ*l antibody mixtures containing 5 ng/*μ*l anti-GST-XL665 (Cisbio China, Shanghai, China) and 0.0225 ng/*μ*l anti-pATF2-EuK (Cisbio China, Shanghai, China) were used at room temperature for 1 h to stop the enzymatic reaction. The OD of drugs' IC_50_ at 665 nm/620 nm was detected with a multimode microplate reader (Tecan Trading AG, Mannedorf, Zurich, Switzerland) (a drug's IC_50_ value signifies the potency of inhibition based on the concentration of inhibitor where 50% inhibition is reached).

### Establishment and monitoring of an intratibial mouse model of breast cancer

Forty female BALB/c-nu/nu mice (4–5 weeks old) were obtained from the Shanghai Slac Laboratory Animal Company (Slac, Shanghai, China). Animals acclimatized for 7 days in plastic-isolator cages before drug intervention were fed with commercial food and water within specific pathogen-free conditions and housed in 12 h dark–light cycles. Before aseptic operations in a laminar-flow hood, animals were sedated by general anesthetization with intraperitoneal ketamine. According to previously well-established records,^59, 71^ 50 *μ*l of bone-targeting MDA-MB-231SArfp cells at a concentration of 5 × 10^6^/ml were injected into the right hind limb of nude mice with an equal volume of phosphate-buffed saline (PBS) injected into the left hind limb as control. Then, mice were randomly assigned to one of four groups (10 nude mice per group). Three days after injection, animals in each group were administered with 100 *μ*l of the relevant reagents via injection (intraperitoneal) (vehicle: PBS, five times a week; Pl: 4 mg/kg body weight, five times a week; Za: 100 *μ*g/kg body weight, two times a week; Syn: 4 mg/kg body weight of PL solution five times a week plus an equal volume of 100 *μ*g/kg body weight of ZA solution two times weeks a week) for up to 6 weeks.

The article "Structural simulation of adenosine phosphate via plumbagin and zoledronic acid competitively targets JNK/Erk to synergistically attenuate osteoclastogenesis in a breast cancer model" was retracted in 2019. Reasons: errors in the images; unreliable data; unreliable images.

Weekly, IVIS imaging (Xenogen, Hopkinton, MA, USA) of the growth of MDA-MB-231SArfp cells within the bone was conducted in each animal. Additionally, tumor size and fluorescence intensity were measured according to methods reported previously.^59^ No fatalities were observed after tumor cell implantation or drug administration, and the mice maintained regular activity throughout the duration of the experiment.

### Evaluations of X-ray and *μ*CT scanning

Osteolytic lesions induced by breast cancer were measured by X-ray radiography (Faxitron, Tucson, AZ, USA) and *μ*CT scanning (*μ*CT 40; Scanco, Zurich, Switzerland) as described previously.^59, 72^ Specifically, nude mice from the various groups were anesthetized and the destruction of tibiae was evaluated with digital radiographic imaging. The integrity of knee-joint architecture as well as the extent of bone erosion after various treatments was compared radiographically. Then, animals were killed and the harvested tumor-bearing tibiae were fixed in 4% paraformaldehyde (pH 7.4). For further *μ*CT tomography, representative tissues were scanned at a resolution of 10 *μ*m with the following parameters: X-ray voltage, 70 kV; electric current, 114 *μ*A. Relevant bone volume fractions (BV/TV) of trabecular and cortical data were obtained.

### H&E staining and immunohistochemistry for RFP

After *μ*CT tomography, representative tumor-bearing tibiae were decalcified, paraffin embedded and sectioned. For H&E staining, sections were stained with H&E using conventional procedures. For immunohistochemical staining, antigen retrieval was performed with trypsin (Mainxin, Fuzhou, China) and endogenous peroxidase activity was blocked with hydrogen peroxide (Mainxin). Then, sections were immersed in corresponding anti-RFP primary antibody and further incubated with second antibody and DAB dye (Mainxin). Hematein was used for staining nuclei. Five random fields of a tumor-bearing area in a representative section of each specimen were imaged, and quantification was accomplished using Image-Pro Plus software (Media Cybernetics, Bethesda, MD, USA).

### Ki-67 immunohistochemistry and TUNEL staining

The proliferative rate of tumor cells was evaluated immunohistochemically based on the expression of Ki-67. Immunohistochemical methods were similar to those above but used an anti-Ki-67 primary antibody. Additionally, the rate of tumor cell apoptosis was determined using the TUNEL assay with the In Situ Cell Death Detection Kit (Roche, Basel, Switzerland) according to the manufacturer's guidelines. Five random fields of a tumor-bearing area in a representative section of each specimen were imaged, and quantification was accomplished using Image-Pro Plus software (Media Cybernetics).

The article "Structural simulation of adenosine phosphate via plumbagin and zoledronic acid competitively targets JNK/Erk to synergistically attenuate osteoclastogenesis in a breast cancer model" was retracted in 2019. Reasons: errors in the images; unreliable data; unreliable images.

### TRAcP staining

Sections were deparaffinized and dehydrated. A commercial TRAcP (387A-1KT; Sigma-Aldrich) was used to stain the TRAcP-positive multinucleated osteoclasts on the bone surface following recommended procedures. The percentage of TRAcP-positive osteoclasts was calculated in five random fields of each section using Image-Pro Plus software (Media Cybernetics).

### Statistical analysis

Data were analyzed with SPSS 13.0 software (Statistical Package for the Social Sciences, Chicago, IL, USA) and presented as the mean±S.D. One-way analysis of variance was used to determine statistically significant differences between various groups. A *P*-value of <0.05 was considered significant.

## Figures and Tables

**Figure 1:** Synergistic inhibition of cell viability on RAW264.7 osteoclast precursor cells via combined treatment with PL and ZA. (**a** and **b**) The growth suppression of RAW264.7 cells after individual treatment with PL (**a**) or ZA (**b**) for 24, 48, 72 and 96 h. (**c**) Combined cytotoxicity after administration with varying ZA concentrations and PL at 0, 2.5, 5, 10 and 20 *μ*M for 24, 48, 72 and 96 h. The fold changes were compared between individual ZA treatments with combinatory treatments. (**d**) Combined cytotoxicity after administrations with varying PL concentrations and ZA at 0, 12.5, 25, 50 and 100 *μ*M for 24, 48, 72 and 96 h. The fold changes were compared between individual PL treatments with combinatory treatments. (**e**) Computerized analysis from the Compusyn software demonstrated the synergistic effect of PL with ZA with Fa-CI and Fa-DRI plots, using the method based on the median effect principle of Chou and Talalay. The data are presented as the means±S.D. All experiments were repeated at least three times (*significant difference at *P*<0.1; **significant difference at *P*<0.05)

**Figure 2:** Combined treatment with PL and ZA synergistically inhibits cancer-induced osteoclastogenesis *in vitro*. (**A**a) BMMs were treated with various concentrations of individual or combined PL and ZA plus RANKL for 5 days. TRAcP staining to elucidate osteoclast formation was performed *in vitro*. (b) The number and percentage of TRAcP-positive MNCs in the individual drug groups and the combination groups. (**B**a) hPBMCs were treated with CM from MDA-MB-231 cells containing various concentrations of individual or combined PL and ZA for 21 days. TRAcP staining to elucidate osteoclast formation was performed *in vitro*. (b) The number and percentage of TRAcP-positive MNCs in the individual drug groups and the combination groups. The data are presented as the means±S.D. All experiments were repeated at least three times. Scale bar=250 *μ*m (*significant difference at *P*<0.1; **significant difference at *P*<0.05)

**Figure 3:** Synergistic treatment with PL and ZA suppresses RANKL-induced activation of the NF-*κ*B/MAPK pathways. After starvation treatment containing various drugs, RANKL was added for 20 min to activate osteoclastogenesis-related signaling pathways. (**A**a) The suppressive effects on the NF-*κ*B signaling cascade. (b) Protein expression levels of NF-*κ*B were calculated. (**B**a) The repressive effects on the MAPK signaling pathway. (b) Protein expression levels of MAPK were calculated. The data are presented as the means±S.D. All experiments were repeated at least three times (**significant difference at *P*<0.05)

**Figure 4:** Structural simulation of ANP by the combined drugs competitively targets phosphorylation of JNK/Erk. (**A**a–c) The two-dimensional chemical structural formulas of PL, ZA and ANP. (d and e) The three-dimensional chemical structural formulas of PL, ZA and ANP. (**B**) Molecular docking of the combination of PL and ZA with JNK-1 or Erk-1 kinases. (**C**) Optimization of reaction conditions for enzymatic activity of the JNK-1/Erk-1 proteases. (**D**) HTRF assay of competitiveness of PL and ZA alone against ANP binding to JNK/Erk. (**E**) HTRF assay of competitiveness of the combined drugs against ANP binding to JNK/Erk. (**F**) BMMs were cultured with 30 ng/ml MCSF and 50 ng/ml RANKL with or without the combined drugs. The downstream expression of c-Jun/c-Fos/NFATc-1 was investigated via western blotting. The data are presented as the means±S.D. All experiments were repeated at least three times (**significant difference at *P*<0.05)

**Figure 5:** A schematic diagram of the proposed mechanisms of osteoclastogenesis inhibition by combined treatment of PL with ZA. The combined administration attenuates the expression of p-I*κ*B*α* and p-p65, thus affecting the NF-*κ*B pathways. Additionally, the mixed drugs abrogate JNK/Erk phosphorylation by competing with the affinity of ANP, thereby inhibiting the downstream production of c-Jun/c-Fos/NFATc-1. Taken together, these events contribute to the downregulation of osteoclast survival, proliferation, differentiation and apoptosis

**Figure 6:** Combined treatment with PL and ZA synergistically inhibits the growth of MDA-MB-231SArfp cells in tumor-bearing mice. Tumor-bearing nude mice were treated with vehicle, PL (4 mg/kg), ZA (100 *μ*g/kg) and Syn (4 mg/kg PL plus 100 *μ*g/kg ZA) for 6 weeks. (**A**) Weekly noninvasive IVIS monitoring of MDA-MB-231SArfp cells inoculated in nude mice (**B**a) The fluorescence intensity of tumor cells within the bone microenvironment at different time points. (b) Breast cancer tumor volume in nude mice at different time points. (c) The correlation between tumor fluorescence intensity and tumor volume. The data are presented as the means±S.D. Each group contained 10 animals (**significant difference at *P*<0.05)

**Figure 7:** Combined treatment with PL and ZA synergistically inhibits breast cancer-induced osteolysis *in vivo*. Representative X-ray radiographs (**A**), *μ*CT tomography of whole tibiae (**B**) and tibial trabecular cancellous structures (**C**) in tumor-bearing mice after 6 weeks of treatment. (**D**) Quantitative data from *μ*CT scanning revealing trabecular BV/TV (a) and Cor. BV/TV (b) after treatments with PL, ZA or both. The data are presented as the means±S.D. Each group contained 10 animals. Scale bar=1.0 mm (*significant difference at *P*<0.1; **significant difference at *P*<0.05)

**Figure 8:** *In vivo* potentiated antiosteoclastogenesis and antitumorigenesis through combined treatment with PL and ZA. (**A**) H&E staining of tibia in tumor-bearing mice after 6 weeks of treatment (magnification, × 200, scale bar=50 *μ*m; magnification, × 400, scale bar=25 *μ*m) (**B**a) TRAcP-positive osteoclasts in the tibiae of tumor-bearing mice after 6 weeks of treatment (magnification, × 400, scale bar=25 *μ*m). (b) Histomorphometric quantifications were calculated. (**C**a) Immunohistochemistry for RFP in tumor tissues (magnification, × 200, scale bar=50 *μ*m; magnification, × 400, scale bar=25 *μ*m). (b) Histomorphometric quantifications were calculated. (**D**a) Immunostaining of Ki-67-positive cells in tumor tissues (magnification, × 200, scale bar=50 *μ*m; magnification, × 400, scale bar=25 *μ*m). (b) Histomorphometric quantifications were calculated. (**E**a) Immunohistochemistry indicating TUNEL-positive cells in tumor tissues (magnification, × 200, scale bar=50 *μ*m). (b) Histomorphometric quantifications were calculated. The data are presented as the means±S.D. Each group contained 10 animals (*significant difference at *P*<0.1; **significant difference at *P*<0.05)

The article "Structural simulation of adenosine phosphate via plumbagin and zoledronic acid competitively targets JNK/Erk to synergistically attenuate osteoclastogenesis in a breast cancer model" was retracted in 2019. Reasons: errors in the images; unreliable data; unreliable images.

## Abbreviations

PL: plumbagin
ZA: zoledronic acid
Syn: synergism
ANP: adenosine phosphate
CI: combination index
DRI: drug-reduction index
BMM: bone marrow macrophage
RANKL: receptor activator for nuclear factor-*κ*B ligand
MCSF: macrophage colony-stimulating factor
CM: conditioned medium
hPBMC: human peripheral blood mononucleated cell
TRAcP: tartrate-resistant acid phosphatase
IC_50_: half-maximal inhibitory concentration
NF-*κ*B: nuclear factor-*κ*B
I*κ*B: inhibitor of NF-*κ*B
IKK: I*κ*B kinase
MAPK: mitogen-activated protein kinase
JNK: c-Jun N-terminal kinase
Erk: extracellular signal-regulated kinase
NFATc-1: nuclear factor of activated T cells, cytoplasmic, calcineurin-dependent 1
HTRF: homogeneous time-resolved fluorescence
IVIS: *in vivo* imaging system
CT: computed tomography
BV/TV: bone volume/tissue volume
RFP: red fluorescent protein
TUNEL: transferase-mediated dUTP biotin nick-end labeling
MNC: multinucleated cell
